# Epidemiological Characteristics and Transmissibility of Human Immunodeficiency Virus in Nanning City, China, 2001–2020

**DOI:** 10.3389/fpubh.2021.689575

**Published:** 2021-12-14

**Authors:** Qian Lin, Bin Deng, Jia Rui, Song-Bai Guo, Qingqing Hu, Qiuping Chen, Chi Tang, Lina Zhou, Zeyu Zhao, Shengnan Lin, Yuanzhao Zhu, Meng Yang, Yao Wang, Jingwen Xu, Xingchun Liu, Tianlong Yang, Peihua Li, Zhuoyang Li, Li Luo, Weikang Liu, Chan Liu, Jiefeng Huang, Min Yao, Mengni Nong, Liping Nong, Jinglan Wu, Na Luo, Shihai Chen, Roger Frutos, Shixiong Yang, Qun Li, Jing-An Cui, Tianmu Chen

**Affiliations:** ^1^Development Planning Office, Guangxi Medical University, Nanning, China; ^2^Department of Science and Technology, School of Public Health, State Key Laboratory of Molecular Vaccinology and Molecular Diagnostics, Xiamen University, Xiamen, China; ^3^Department of Mathematics and Data Science, School of Science, Beijing University of Civil Engineering and Architecture, Beijing, China; ^4^Division of Public Health, School of Medicine, University of Utah, 201 Presidents Circle, Salt Lake, UT, United States; ^5^Laboratory Intertryp CIRAD/IRD, Université de Montpellier, Montpellier, France; ^6^Department of Medical Insurance Office, Xiang'an Hospital of Xiamen University, Xiamen, China; ^7^Division of Director's Office, Nanning Municipal Health Commission, Nanning, China; ^8^Department of Nephrology, The Second Hospital of Xiamen Medical College, Xiamen, China; ^9^Department of STD and AIDS Prevention and Treatment, Nanning Center for Disease Control and Prevention, Nanning, China; ^10^Department of Health Emergency, Chinese Center for Disease Control and Prevention, Beijing, China

**Keywords:** human immunodeficiency virus, transmission model, transmissibility, dynamics, acquired immune deficiency syndrome

## Abstract

**Background:** Human immunodeficiency virus (HIV) is a single-stranded RNA virus that can weaken the body's cellular and humoral immunity and is a serious disease without specific drug management and vaccine. This study aimed to evaluate the epidemiologic characteristics and transmissibility of HIV.

**Methods:** Data on HIV follow-up were collected in Nanning City, Guangxi Zhuang Autonomous, China. An HIV transmission dynamics model was built to simulate the transmission of HIV and estimate its transmissibility by comparing the effective reproduction number (*R*_*eff*_) at different stages: the rapid growth period from January 2001 to March 2005, slow growth period from April 2005 to April 2011, and the plateau from May 2011 to December 2019 of HIV in Nanning City.

**Results:** High-risk areas of HIV prevalence in Nanning City were mainly concentrated in suburbs. Furthermore, high-risk groups were those of older age, with lower income, and lower education levels. The *R*_*eff*_ in each stage (rapid growth, slow growth, and plateau) were 2.74, 1.62, and 1.15, respectively, which suggests the transmissibility of HIV in Nanning City has declined and prevention and control measures have achieved significant results.

**Conclusion:** Over the past 20 years, the HIV incidence in Nanning has remained at a relatively high level, but its development trend has been curbed. Transmissibility was reduced from 2.74 to 1.15. Therefore, the prevention and treatment measures in Nanning City have achieved significant improvement.

## Introduction

In 1938, HIV was isolated for the first time (1). HIV attacks the body's immune system, leading to a decrease in the CD4^+^T lymphocytes in the body (2, 3). The early clinical symptoms of patients with HIV infection patients are fever, myalgia, and other cold-like symptoms. Patients who are later diagnosed with HIV have a partial or complete loss of immune function as the number of CD4^+^T cells decrease, and opportunistic infections and tumors occur. Therefore, more patients with AIDS die from co-infection of other diseases (4, 5). HIV is divided into two types: HIV-1 and HIV-2. HIV-1 is the most widely spread globally, while HIV-2 is concentrated in western and central Africa (1, 6).

According to the WHO report, since the start of the HIV epidemic, 76 million people have been infected worldwide, and 33 million people have died. However, as of 2019, 38 million people are still infected with HIV (7). Since 2010, most new HIV infections have been reported in Asia (8). Although the prevalence of HIV in the Asia-Pacific region remains relatively low (about 15.35%) (9), as of 2020, only three countries have achieved the 90–90–90 goals (90% of people with HIV diagnosed, 90% on antiretroviral therapy, 90% virologically suppressed) in Asia, excluding China (10). In China, the HIV epidemic started later. The first HIV case in China was reported in 1985, and systematic prevention and control measures have been adopted since 1986 (11). Although the total HIV detection rates in China increased 4-fold from 2009 to 2018, and the number of people with HIV dropped from 0.11 to 0.06%, there were 861,042 people infected with HIV at the end of 2018 (12). Guangxi Zhuang Autonomous Region ranked third among all provinces in China for HIV cases, with an HIV infection rate of 0.13% among the general population. The HIV epidemic was frequent in middle-aged and elderly men over the age of 50. Most people with HIV infection were infected through heterosexual contact (13, 14).

In China, the main routes of HIV transmission are sexual transmission, blood transmission, and mother-to-child transmission (15). Early in the epidemic in China, the proliferation of drug trade led to the spread of HIV, but with the advancement of antiretroviral treatment (ART) and controlling illegal activities such as drugs and blood buying, the rate of mother-to-child transmission and blood transmission has been reduced. After 2006, sexual transmission has become the main transmission route as drugs and blood sales were restricted. HIV transmission through sex work has gradually become the mainstream source. Additionally, in recent years, the HIV transmission rate among men who have sex with men (MSM) has risen rapidly (16, 17).

Existing HIV research mainly discusses two aspects: virology and epidemiology. Most existing studies focus on virology, exploring microscopic topics, such as the virus structure and pathogenesis of HIV (3, 18, 19). There were relatively few epidemiological studies, mainly focusing on the effectiveness of new treatment drugs and ART (20, 21), as well as the prediction and analysis of HIV transmission in different populations (22, 23). In addition, there are few studies on the transmissibility of HIV, and very few obtained HIV transmission rates through cohort follow-up (24, 25). Mathematical models were the most common method to study HIV transmission. The validity of the established model was proven by deriving mathematical deduction (26) or using statistical models to analyze the influencing factors of HIV (27, 28). However, the mathematical model was used to fit real data, calculate the transmissibility of HIV, and evaluate the impact of HIV (29, 30). In general, most studies on the dynamics of HIV transmission in China were based on mathematical deductions and demonstrations in terms of model stability and parameter values (31, 32). For example, some researchers have used dynamic and stochastic models to predict the effectiveness of various interventions in China or established a transmission dynamics model to calculate the transmission rate between different ages (33, 34). Few studies can apply the model to a specific area of China or within a certain period from the perspective of public health and apply the model to practice, however. In epidemiology, the basic reproduction number (*R*_0_) was used to determine whether the disease can spread continuously. *R*_0_ was defined as the average number of secondary infections produced by an infected person in an area where all people are susceptible (35). At present, few studies used *R*_0_ to assess the spread of HIV.

Most studies focused on the spread of HIV within a community or a short period. There were few studies on the spread of HIV within a city for a significantly long time, which does not allow us to discover the difference in trends in disparate times and account for specific prevention and control measures based on those trends. Therefore, this study used the HIV report data of Nanning City from 2001 to 2020 to establish a transmission dynamics model. Based on the epidemic characteristics of Nanning City and the HIV transmission characteristics, this model was fitted to report data, calculate HIV transmissibility in Nanning City, and evaluate the effect of local prevention and control. This study also provided a theoretical basis for achieving the 95–95–95 target (95% of people with HIV diagnosed, 95% on antiretroviral therapy, 95% virologically suppressed) in 2035.

## Methods

### Study Area

Nanning City is located in the southern region of China, adjacent to the Socialist Republic of Vietnam. As of February 2021, Nanning had a total area of 22,112 square kilometers and a permanent population of 7,344,800 people.

### Data Collection

The HIV data from January 2001 to May 2020 were collected by the Nanning Centres for Disease Control (CDC), which included the monthly distribution of cases and the date of death. The population, birth rates, and death rates from 2001 to 2019 were collected from the Nanning Statistics Bureau.

Three methods were used by Nanning to conduct the under-reporting of HIV epidemic reports: (1) national data quality verification was conducted from July to August every year; (2) the Nanning Municipal Health Commission entrusted the Municipal Center for Disease Control (CDC) and Prevention every year to organize and carry out spot checks on HIV reports of medical institutions in the city; (3) the Sexually Transmitted Disease and AIDS Prevention and Control Department of the Municipal CDC conducted an HIV epidemic report work inspection twice a year. We inspected the collected data by checking the positive result registry from the HIV screening laboratory of the medical institution and compared the records with the national HIV epidemic report database. If the record was in the registry but not entered in the national database, it was classified as underreporting. False report rate was defined as the number of false reports divided by the total number reported (confirmed HIV positive).

### Establishment of HIV Transmission Dynamics Model

Based on the epidemic characteristics of HIV, we built the Susceptible-Exposed-Untested HIV infection-Tested HIV infection-Dead (SEITD) model. In the SEITD model, we regarded *S* as the suspectable population, *E* as someone who is exposed to HIV, *I* as individuals who have HIV but were not tested, *T* as individuals who have HIV and were tested, and *D* as individuals who died from HIV. Those tested people were HIV-infected and patients with AIDS. The difference between the patients with HIV and those with AIDS is that they are in different stages of the disease. The persons infected with HIV refer to those who have HIV in their bodies but still live normally, while patients with AIDS refer to individuals with HIV infection whose immune function has been affected and may be at risk of opportunistic infection. The definitions of these variables are listed in Table 1 and the model structure is shown in Figure 1. The SEITD model was based on the following assumptions:

1) All newborns are susceptible, birth rate (*br*); death rate (*dr*); and *N* is a stable constant for the whole population.
2) *S* are infected through contact with *I*, and the transmissibility is β. It is assumed that the transmissibility of *T*_1_ and *T*_2_ is κ_1_ and κ_2_ times that of *I*, and that the transmissibility of *T*_2_ is higher than *T*_1_, then the κ_2_ < κ_1_.
3) The latent period of *E* is ω, the latent period is the time from HIV exposure to the acute phase of HIV. According to the literature (4, 36), the latent period is 2–6 weeks, so ω=4 weeks.
4) Among the *I*, after diagnosis, a percentage of people with the infection will be diagnosed as *T*_1_, and this percentage is *p*. Because *I* will become *T*_2_ after an average incubation period, the other portion of people infected will be diagnosed as *T*_2_, and this percentage is (1–*p*). Additionally, for *T*_1_ and *T*_2_, the diagnosis has time lag α, but for patients with AIDS, the time lag should add to the incubation period, so the calculation formula of δ is as follows: δ = α + incubation period.
5) For *T*_1_ and *T*_2_, the fatality rates were set as *f*_1_ and *f*_2_, respectively in this study.

**Table 1:** Variables and definition of the structure of the HIV transmission dynamics model.

**Variables**	**Definition**
S	Susceptible population
E	Exposed population
I	Untested HIV-infected
T_1_	Tested HIV-infected
T_2_	Tested AIDS patient
D_1_	Dead of HIV infection in tested HIV-infected
D_2_	Dead of HIV infection in tested AIDS patient

**Figure 1:** The structure of HIV transmission dynamics model.

The differential equation of the SEITD model is expressed as follows:


$$\begin{array}{l} \;\frac{dS}{dt}=b_{r}N{-d}_{r}S-\beta S\left(I+K_{1}T_{1}+K_{2}T_{2}\right)\\ \;\frac{dE}{dt}=\beta S\left(I+K_{1}T_{1}+K_{2}T_{2}\right)-d_{r}E-\omega E\\ \;\frac{dI}{dt}=\omega E-d_{r}I-p\alpha I-\left(1-p\right)\delta I\\ \frac{dT_{1}}{dt}=p\alpha I-d_{r}T_{1}-f_{1}T_{1}\\ \frac{dT_{2}}{dt}=\left(1-p\right)\delta I-d_{r}T_{2}-f_{2}T_{2}\\ \frac{dD_{1}}{dt}=f_{1}T_{1}\\ \frac{dD_{2}}{dt}=f_{2}T_{2} \end{array}$$

The left side of the equation is represented as the instantaneous change of speed of *S, E, I*, *T*_1_, *T*_2_, *D*_1_, and *D*_2_ at time *t*.

### Parameter Estimation

In this model, the main parameters included the proportion of the HIV-infected individuals (*p*), HIV latent period (ω), the fatality rate of the HIV-infected (*f*_1_), the fatality rate of the patients with AIDS (*f*_2_), birth rate (*br*), death rate (*dr*), and the diagnosis time lag of the HIV-infected (α) were collected from HIV follow-up data. The diagnosis time lag of patients with AIDS (δ) is calculated by α and an average incubation period of HIV. HIV transmissibility (β) needs to be fitted based on the HIV-reported data. We carried out a descriptive analysis for *f*_1_, *f*_2_, *p*, and α. The value of α was 0.47 months, and according to the literature (4, 36, 37), the average incubation period of HIV was 4.5 years, so δ is 54.47 months, and the latent period was 2–6 weeks, so ω was 0.94 months. Although the *br, dr*, *f*_1_, *f*_2_, and *p* have different values in different stages, we still decided to take their average values and utilize them in the model. Further details on the definition and value of the parameters were provided in Tables 2, 3.

**Table 2:** Definition and value of parameters in HIV transmission dynamics model.

**Parameters**	**Definition**	**Value**	**Unite**	**Range**	**Methods**
β	HIV transmissibility	–	–	–	Model fitting
*p*	Proportion of the HIV- infected	0–0.46	1	0.4–0.52	Data collection
ω	Latent period	0.94	Months	0.47–2.8	References (4, 36)
κ_1_	Transmissibility coefficient of the HIV-infected	0.1	1	–	Hypothesis
κ_2_	Transmissibility coefficient of AIDS patients	0.9	1	–	Hypothesis
α	Period from onset time to diagnosis as the HIV-infected	0.47	Months	0–200	Data collection
δ	Period from onset time to diagnosis as the AIDS patients	54.47	Months	0–254	Data collection and Reference (37)
*f*_1_	Fatality rate of the HIV-infected	0.035	1	0.00059–0.06060	Data collection
*f*_2_	Fatality rate of AIDS patients	0.033	1	0.00676–0.04540	Data collection
*b*_*r*_	Birth rate	0.00081	1	0.00047–0.00127	Statistical Yearbook of Nanning City
*d*_*r*_	Death rate	0.00021	1	0.00011–0.00047	Statistical Yearbook of Nanning City

**Table 3:** The value of parameters of *br, dr*, *f*_1_, *f*_2_ and *p* in detail.

**Parameters**	**Stages**	**Value**	**Units**
*b*_*r*_	January 2001 to March 2005	0.000637	1
	April 2005 to April 2011	0.001159	1
	May 2011 to December 2019	0.000693	1
*d*_*r*_	January 2001 to March 2005	0.000226	1
	April 2005 to April 2011	0.000326	1
	May 2011 to December 2019	0.000157	1
*f*_1_	January 2001 to March 2005	0.057143	1
	April 2005 to April 2011	0.046396	1
	May 2011 to December 2019	0.012909	1
*f*_2_	January 2001 to March 2005	0.040650	1
	April 2005 to April 2011	0.038671	1
	May 2011 to December 2019	0.029299	1
*p*	January 2001 to March 2005	0.44	1
	April 2005 to April 2011	0.39	1
	May 2011 to December 2019	0.49	1

The basic reproduction number (*R*_0_) is often used when the disease occurs naturally. If *R*_0_ is greater than 1, it is sufficient to maintain disease transmission; if *R*_0_ is less than 1, it cannot cause disease transmission. But the occurrence and development of the disease are often affected by many factors and *R*_0_ can only represent the initial transmissibility of a disease. Our research period is large, so the effective reproduction number (*R*_*eff*_) represents the transmissibility of diseases in different periods. Therefore, the *R*_*eff*_ was used to replace *R*_0_. This study used *R*_*eff*_ to estimate the transmissibility of HIV and the formula of *R*_*eff*_ was derived according to the second-generation matrix method; the formula is as follows:


$$\begin{array}{l} f=\left(\begin{array}{c} \beta S\left(I+\kappa_{1}T_{1}+\kappa_{2}T_{2}\right)\\ 0\\ 0\\ 0 \end{array}\right) \end{array}$$

$$\begin{array}{l} v=\left(\begin{array}{c} d_{r}E+\omega E\\ -\omega E+d_{r}I+p\alpha I+\left(1-p\right)\delta I\\ -p\alpha I+d_{r}T_{1}+f_{1}T_{1}\\ -\left(1-p\right)\delta I+d_{r}T_{2}+f_{2}T_{2} \end{array}\right)\\ F=\left(\begin{array}{cccc} 0 & \beta brN/dr & \beta brN/dr\kappa_{1} & \beta brN/dr\kappa_{2}\\ 0 & 0 & 0 & 0\\ 0 & 0 & 0 & 0\\ 0 & 0 & 0 & 0\\ \; \end{array}\right)\\ V=\left(\begin{array}{cccc} d_{r}+\omega & 0 & 0 & 0\\ -\omega & d_{r}+p\alpha +\left(1-p\right)\delta & 0 & 0\\ 0 & -p\alpha & d_{r}+f_{1} & 0\\ 0 & -\left(1-p\right)\delta & 0 & d_{r}+f_{2}\\ \; \end{array}\right) \end{array}$$

$$\begin{array}{l} V^{-1}=\\ \left(\begin{array}{cccc} \frac{1}{d_{r}+\omega } & 0 & 0 & 0\\ \frac{\omega }{\left(d_{r}+\omega \right)\left[d_{r}+p\alpha +\left(1-p\right)\delta \right]} & \frac{1}{d_{r}+p\alpha +\left(1-p\right)\delta } & 0 & 0\\ \frac{\omega p\alpha }{\left(d_{r}+f_{1}\right)\left(d_{r}+\omega \right)\left[d_{r}+p\alpha +\left(1-p\right)\delta \right]} & \frac{p\alpha }{\left(d_{r}+f_{1}\right)\left[d_{r}+p\alpha +\left(1-p\right)\delta \right]} & {\frac{1}{d_{r}+f}}_{1} & 0\\ \frac{\omega \left(1-p\right)\delta }{\left(d_{r}+f_{2}\right)\left(d_{r}+\omega \right)\left[d_{r}+p\alpha +\left(1-p\right)\delta \right]} & \frac{\left(1-p\right)\delta }{\left(d_{r}+f_{2}\right)\left[d_{r}+p\alpha +\left(1-p\right)\delta \right]} & 0 & \frac{1}{d_{r}+f_{2}}\\ \; \end{array}\right)\\ R_{eff}=\rho \left(FV^{-1}\right)=\frac{\beta \omega b_{r}N}{d_{r}\left(d_{r}+\omega \right)\left[d_{r}+p\alpha +\left(1-p\right)\delta \right]}\\ \;+\frac{\beta b_{r}N\kappa_{1}\omega p\alpha }{d_{r}\left(d_{r}+f_{1}\right)\left(d_{r}+\omega \right)\left[d_{r}+p\alpha +\left(1-p\right)\delta \right]}\\ \;+\frac{\beta b_{r}N\kappa_{2}\omega \left(1-p\right)\delta }{d_{r}\left(d_{r}+f_{2}\right)\left(d_{r}+\omega \right)\left[d_{r}+p\alpha +\left(1-p\right)\delta \;\right]} \end{array}$$

### Method and Data Analysis

Based on different epidemic characteristics, the HIV epidemic was divided into three stages: the rapid growth period (from January 2001 to March 2005); the slow growth period (from April 2005 to April 2011); and the plateau (from May 2011 to December 2019) (Figure 2). The SEITD model was used to fit the HIV-reported data using the Least Mean Squares in Berkeley Madonna and calculate the transmissibility in these stages. The fitting database, as reported by the Nanning Centre for Disease Control and Prevention from January 2001 to May 2020, included 22,698 people with HIV infection 46.57% of those were HIV-infected people and 53.43% were patients with AIDS. Afterward, we used the transmissibility at each stage, calculated by the SEITD model to simulate the HIV prevalence curve at each stage without intervention. The effect of prevention measures on HIV can be estimated by comparing the epidemic curves between stages of the simulated epidemic and reported epidemic. The evaluation index includes the total number of cases, total attack rate, peak time, and peak attack rate.

**Figure 2:** The number of cases and incidence rate of HIV in Nanning from 2001 to 2020.

We used EXCEL2019 (Microsoft Corporation, Washington, USA) to preliminarily process and chart the data, and the central trend was described by the median. IBM SPSS (version 21.0.0) (IBM, New York, USA) was used for the statistical analysis and *P* < 0.05 indicated that the difference was statistically significant. Berkeley Madonna (version 8.3.18) was used to fit the existing data and models to simulate the HIV epidemic.

## Results

### Epidemic Characteristics of HIV

The HIV follow-up data from Nanning City were collected from January 2001 to May 2020, with a total of 22,697 cases. Among these, 12,126 were patients with AIDS, and 10,571 were patients with HIV infection. After 20 years of follow-up, 7,068 patients with HIV/AIDS died, including 2,693 HIV-infected and 4,376 patients with AIDS.

Overall, as shown in Figures 2, 3, the HIV epidemic trend in Nanning City showed three stages. In the first stage, the monthly incidence rate of HIV steeply rose from 1.58 (per 10,000) to 1.85 (per 10,000) in 50 months. Before 2004, there were basically no reports of HIV cases in January and February, and there was no obvious pattern in case reports. Since 2004, the number of cases per quarter has gradually increased and peaked in March 2005. At this stage, there was no obvious trend the fatality rate.

**Figure 3:** The number of deaths and fatality rate of HIV in Nanning for twenty years.

In the second stage, although the monthly HIV incidence rate steadily rose, there was a sharp increase in the number of cases in the spring of 2005. The number of cases in one month increased from an average of 10 in the first stage to 78 in May 2005. This suggested that the prevalence of HIV in Nanning was gradually increasing. The fatality rate also began to rise gradually in April 2005, with an average fatality rate of 16 people, see Figures 2, 3.

In the third stage, there was still a slight upward trend in 2011, resulting in an average monthly incidence of 151 people. In 2012, the developing trend of HIV in Nanning had gradually stabilized, and the incidence rate had stabilized at 2.02 (per 10,000), see Figure 2. As shown in Figure 3, from the third phase (October 2011), the overall HIV mortality rate in Nanning City had developed an overall declining trend. From 2012 to 2016, there was a sudden increase in the yearly fatality rate.

From January 2001 to May 2020, 22697 HIV-prevalent cases were reported by the NCDC. As shown in Figure 4, the distribution of HIV in Nanning City has gradually expanded over time. In the first stage, the number of HIV reports in Nanning City gradually increased. Until 2005, all areas of Nanning City had reported HIV cases, but there was little difference in incidence rates between regions. Since the second phase, the number of reported cases in the Nanning City suburbs (Heng County, Binyang County, Xixiangtang District, etc.) has been increasing yearly. The regional distribution showed that the incidence in the North and South was less and the incidence in the East and West was higher. At the beginning of the third phase (2011–2013), the number of reported cases in Heng County, Mashan County, and Binyang County peaked. From the third phase, confirmed HIV cases have also been reported in the northern areas of Nanning City (Mashan County and Shanglin County). From 2001 to 2014, the number of yearly reported HIV cases in Nanning City rose from 96 to 1674; but from 2015 to 2019, the HIV prevalence in Nanning City stabilized. All reported HIV prevalence cases in Nanning City were mainly concentrated in Heng County, Binyang County, Xixiangtang District, Longan County, Jiangnan District, Mashan County, and Shanglin County. Among these areas, Heng County was the most affected area, with 5,097 cumulative cases over the years, accounting for 22.46% of all cases. This was followed by Binyang County, which accounted for 11.51%. Yongning District and Liangqing District have been at a low level, with a cumulative number of cases of 705 and 982 over the years, respectively.

**Figure 4:** The distribution by place of HIV in Nanning for 20 years (The signal of the red point represents the site of Nanning city in China).

Among the 22,697 HIV-infected persons, 16,910 (74.5%) were men and 5,787 (25.5%) were women. According to Figure 5 and Table 4, it can be found that in the past 20 years, the incidence of HIV in both men and women in Nanning City increased with time, but the incidence in men was consistently higher than women, and the difference between men and women was statistically significant (*P* < 0.05). At different stages, the gender composition ratio of confirmed HIV cases in Nanning City is also significantly different (*P* < 0.05). Though most cases were men, the proportion of women with HIV has increased over time from 15.64% in the first stage to 33.54% in the third stage. At different stages, there are differences in the composition ratio of HIV-infected persons' marital status. In the first stage, unmarried people with HIV infection accounted for the majority (35.99%), but from the second stage, most HIV-infected people were married.

**Figure 5:** The distribution by sex of HIV in Nanning from 2001 to 2019.

**Table 4:** The distribution by people of HIV in three stages in Nanning from January 2001 to May 2020.

**Factors**	**Stage 1** ^**#**^		**Stage 2** ^**#**^		**Stage 3** ^**#**^	
	**Number of cases**	**Percentage (%)**	**Number of cases**	**Percentage (%)**	**Number of cases**	**Percentage (%)**
Sex^*^	614	100.00%	5,652	100.00%	16,431	100.00%
Male	518	84.36%	4,088	72.33%	11,846	12,304
Female	96	15.64%	1,564	27.67%	3,996	4,127
Matrimony^*^	614	100.00%	5,652	100.00%	16,431	100.00%
Married	190	30.94%	3,551	62.83%	9,122	55.52%
Unmarried	221	35.99%	1,277	22.59%	4,132	25.15%
Divorced or widowed	38	6.19%	606	10.72%	3,157	19.21%
Unknow	165	26.87%	218	3.86%	20	0.12%
Age^*^	614	100.00%	5,652	100.00%	16,431	100.00%
< 1	0	0.00%	0	0.00%	2	0.01%
1–	2	0.33%	49	0.87%	41	0.25%
10–	15	2.44%	46	0.81%	208	1.27%
20–	235	38.27%	1,054	18.65%	2,218	13.50%
30–	245	39.90%	1,676	29.65%	2,567	15.62%
40–	87	14.17%	979	17.32%	2,828	17.21%
50–	22	3.58%	666	11.78%	3,029	18.43%
60–	5	0.81%	629	11.13%	3,429	20.87%
70–	3	0.49%	481	8.51%	1,826	11.11%
80–	0	0.00%	71	1.26%	273	1.66%
90–	0	0.00%	1	0.02%	10	0.06%
>100	0	0.00%	0	0.00%	0	0.00%
Occupation^*^	614	100.00%	5,652	100.00%	16,431	100.00%
Technicist	207	33.71%	1,210	21.41%	2,291	13.94%
Farmar	121	19.71%	2,755	48.74%	10,183	61.97%
Civilian staff	13	2.12%	117	2.07%	327	1.99%
Business services	29	4.72%	212	3.75%	640	3.90%
Student	4	0.65%	78	1.38%	486	2.96%
Worker	21	3.42%	421	7.45%	612	3.72%
Military	0	0.00%	0	0.00%	0	0.00%
Unclassified	219	35.67%	849	15.02%	1,892	11.51%
Degree of education^*^	399	64.98%	5,432	96.11%	16,431	100.00%
Junior college and above	10	1.63%	224	3.96%	1,817	11.06%
High school	23	3.75%	561	9.93%	1,748	10.64%
Junior high school	267	43.49%	2,438	43.14%	5,624	34.23%
Primary school	93	15.15%	1,894	33.51%	6,462	39.33%
Illiteracy	6	0.98%	315	5.57%	780	4.75%

# *Stage 1: rapid growth period (from January 2001 to March 2005); Stage 2: slow growth period (from April 2005 to April 2011); Stage 3: the plateau (from May 2011 to December 2019)*.

* *The difference in the composition ratio of the factors at different stages is statistically significant (P < 0.001)*.

Overall, most of the people with HIV infection were from 30 to 70 years old, with a total of 19,663 (78.80%) cases. Similarly, the age composition of people with HIV infection was different at different stages (*P* < 0.001). In general, as time increased, people with HIV infection in Nanning City gradually concentrated in the middle-aged and elderly people over 50 years old. In the first stage, most of the infected people were concentrated in young people aged 20–30 (78.17%). In the second and third stages, most of the people with HIV infection were concentrated in middle-aged people aged 30–60, accounting for 69.89 and 72.14%, respectively. In terms of occupation, the occupational composition of people with HIV infection between the three stages was also different (*P* < 0.001). In the first stage, the main sources of HIV-infected persons in Nanning City were technicians (33.71%) and farmers (19.71%). In the second and third stages, farmers became the main population of HIV transmission in Nanning City, accounting for 48.74 and 61.97%, respectively. For people living with HIV at different stages in Nanning City, education level was one of the factors that influenced notable differences (*P* < 0.001). Nanning City has gradually improved the education level survey of people with HIV infection and the proportion of the surveyed population has increased from 64.98% in the first stage to 100% in the third stage. However, the education level of people with HIV infection in the three stages was concentrated in junior high school and below. Compared to the first stage, the proportion of people with HIV infection with junior high school and above has increased from 3.75 to 11.06%, more details are shown in Table 4.

### Descriptive Analysis of Parameters

The diagnosis time lag (α) gradually decreased with the increase in time, and the distribution gradually stabilized after 11 years and the third stage, as shown in Figure 6. For the fatality rate of HIV-infected (*f*_1_), there was no uniform change in all stages. The distribution of the second and third stages was stable, but the case fatality rate increased gradually in the third stage (Figure 7A). The mortality rate of AIDS (*f*_2_) and the proportion of HIV-infected (*p*) changed in the same way, declining with the increase in time in all stages. The distribution stabilized in the third stage, see Figures 7B,C.

**Figure 6:** Time of diagnosis in different years and stages. **(A)** The diagnosis time changes from 2001 to 2020; **(B)** the diagnosis time changes in different stages.

**Figure 7:** Parameter of *f*_1_, *f*_2_, and *p* in three stages. **(A)** The fatality rate of HIV-infected (*f*_1_) in different stages; **(B)** the fatality rate of AIDS patient (*f*_2_) in different stages; **(C)** the proportion of HIV-infected (*p*) in different stages.

### Curve Fitting and Calculation of Transmissibility

The fitting results of the model and the original incidence rate of HIV in Nanning are shown in Figures 8, 9A. The model-fitting results were satisfactory (*R*^2^ = 0.82, *P* < 0.001), and showed that the *R*_*eff*_ of the first, second, and third stage was 2.74, 1.62, and 1.15, respectively.

**Figure 8:** The Susceptible-Exposed-Untested HIV infection-Tested HIV infection-Dead (SEITD) model fitting result of HIV reported data of 2001–2019 in Nanning City.

**Figure 9:** The result of simulation prevention and control effect of HIV in Nanning during the twenty years. **(A)** The result of the model fitted and different stage in the development of HIV, Rapid growth period: from January 2001 to March 2005; Slow growth period; from April 2005 to April 2011; Plateau: from May 2011 to December 2019; **(B)** the result of the simulated trend by using the transmissibility of rapid growth period without interventions; **(C)** the result of the simulated trend by using the transmissibility of slow growth period in the condition of without interventions in the second stage but taking interventions in the rapid growth period.

The results suggested that, compared with the reported data, the first stage had a *R*_*eff*_ of 2.74. Based on the *R*_*eff*_, the number of people infected with HIV in Nanning will increase just like the trend shown in Figure 9B, by the end of 2019. If no interventions were used in the first stage, the number of HIV cases within 20 years would have increased from 22,697 to 7,047,289. This confirms that the interventions in Nanning City have been effective, making the reported cases decreased by 99.67%. In the second stage with a *R*_*eff*_ of 1.62, if we used the interventions in the first stage but not in the second stage, there would be more people with HIV infection by the end of 2019, as shown in Figure 9C. The reported data, however, was not as high as the simulated data, which suggests that the interventions in those stages had a significantly positive effect.

### Sensitivity Analysis

In the SEITD model, κ_1_ and κ_2_ were our assumptions. Therefore, a sensitivity analysis of both parameters showed that the value of κ_1_ kept decreasing and the value of κ_2_ kept increasing. Therefore, the HIV transmissibility at different stages in Nanning City will gradually decrease, and the *R*_*eff*_ will eventually drop below 1, which suggests that HIV will no longer be transmitted in Nanning City (Figure 10).

**Figure 10:** The sensitivity analysis of κ_1_ (*κ_1_: transmissibility coefficient of the HIV-infected, κ_1_ + κ_2_ = 1).

## Discussion

In this study, we used the 20-year HIV report data and transmission characteristics of Nanning City to establish a more realistic SEITD transmission dynamics model and we calculated the HIV transmissibility of Nanning in different periods through model fitting and simulation and evaluated the effect of HIV prevention and control measures in Nanning over 20 years.

The time distribution of HIV in Nanning showed that the reported HIV incidence rates and fatality rate before 2004 had no obvious pattern and in the first stage, the transmissibility of HIV in Nanning was high (*R*_*eff*_ = 2.74), which may be attributed to poor data collection and the lack of systematic HIV prevention and control measures in Nanning (38). The distribution of *f*_1_, *f*_2_, *p*, and α in the first stage reflects this. In 2005, the number of reported cases began to rise slowly and steadily, and transmissibility decreased (*R*_*eff*_ = 1.62), which may be due to the implementation of the AIDS voluntary testing and counseling program in September 2004 by the National Health Commission of the People's Republic of China. The Guangxi Zhuang Autonomous Region also publicized the AIDS counseling hotline in January 2005 (38, 39). This intervention may have improved the detection rate of people with HIV infection, allowing more people with HIV infection to be discovered and access treatment. HIV transmissibility decreases with the treatment of ART drugs, which will reduce the rate of HIV transmission in Nanning City (40). In the third stage, although the number of HIV cases was at a high level and transmissibility decreased (*R*_*eff*_ = 1.15), the development trend was relatively stable, which may have been due to the “Twelfth Five-Year Plan for Containment and Prevention of AIDS in China” issued in 2012. With the development of AIDS education, combating the sex trade, and quickly establishing a rescue system, the prevention and management of HIV in Nanning City has achieved a level of success (38, 41). With the implementation of HIV education work, general awareness of HIV will increase, which may influence the general population to be more active in prevention and management efforts. This will also improve the rate of condom use. Individual behaviors will reduce the population's susceptibility and reduce the speed of HIV transmission (10, 42). From 2005 to 2011, the HIV fatality rate in Nanning City was at a high level and slowly increased. This may be because HIV/AIDS was not included in the medical assistance program at that time, which led to the continuous increase in the number of deaths and the fatality rate (43). With the launch of prevention and control work in 2012, the mortality rate of HIV in Nanning has gradually decreased and stabilized in recent years. In the early stage of the third phase, most cases died in the winter. This may have been because the HIV prevention and control system was not perfect at that time, leading to reporting of death information for most cases at the end of the year. Since the inclusion of HIV treatment in the medical aid plan, the sources of HIV infection and the spread of HIV in Nanning City may be reduced (24).

The spatial distribution of HIV in Nanning City showed that cases were mainly distributed in the border areas of Nanning City, such as Heng County, Binyang County, and Xixiangtang District., which are the most serious, but Yongning District and Liangqing District in the south have been at a lower level. This may be because Heng County and Binyang County are closer to Guigang, Laibin, and Liuzhou, which are cities with high HIV incidence rates. In addition, Guangxi Zhuang Autonomous Region and Yunnan Province were on drug trade routes, and border tourism with high population flow may increase the incidence rate of HIV (44, 45).

Over the past twenty years, the distribution of people with HIV in Nanning showed that men were the main infected population and the incidence of HIV in men was higher than in women. This may be due to the main transmission route from drug use to sex, and the rapid development of male-to-male sex transmission in recent years may lead to a greater chance of men being infected with HIV (44). Additionally, more than 36.51% of HIV cases were in men over 50 years old with low educational levels. This may be due to the increased availability of drugs for the treatment of erectile dysfunction in elderly men, incorrect use of condoms, and low HIV education. Therefore, people of older age, low income, and educational levels have become representative of the HIV distribution in Nanning (46). From January 2001 to December 2019, the change in *R*_*eff*_ was consistent with previous studies (47).

In summary, the HIV prevalence in Nanning City mainly rose first and then stabilized, although the *R*_*eff*_ was decreased from 2.74 to 1.15 and the interventions have achieved significant positive effects. The above discussion on the impact of HIV prevention and control measures was from the perspective of the developmental direction of HIV that is most likely to be effective. Specific intervention measures were aimed at the transmission route or source of HIV infection; however, it is necessary to further establish a transmission dynamic model with intervention measures for separate analysis. Although certain interventions have been implemented, the incidence rate of HIV is still high. We suspect that this is because the development trend of HIV has been contained; however, due to the particularity of HIV, there is a lack of medicines or preventive measures, like vaccines, to strictly control spread.

The value of *R*_*eff*_ reminds us that the HIV epidemic still requires interventions to maintain progress, More studies are necessary to address HIV transmission and treatment. To reach the 95–95–95 target by 2035, based on original prevention and control measures the following aspects need to be considered: (1) focus on controlling the spread of HIV among middle-aged and elderly people; (2) strengthen HIV surveillance in urban fringe areas; (3) further popularize HIV prevention and treatment education to people with lower education levels; (4) address opportunities in MSM transmission.

### Limitations

In this study, the data set used was the HIV report card from the NCDC and Prevention from 2001 to 2020. The data collection system was probably imperfect in the early stages, and the data for 2020 included only five months, so it may not be comparable to other years. Furthermore, we built a population-wide HIV transmission dynamics model. This model does not consider differences in behavior, habits, and disposition among individuals. Different age groups have an obvious heterogenicity in the transmission of HIV, but this study did not consider those effects.

## Conclusion

The HIV prevention measures of Nanning City have achieved significant results, which reduced the HIV transmissibility from 2.74 to 1.15, but still maintains a high morbidity rate. Further prevention and control are required.

## Data Availability Statement

The original contributions presented in the study are included in the article/supplementary material, further inquiries can be directed to the corresponding authors.

## Author Contributions

TC, JR, QL, and BD designed the research. BD, JR, QL, S-BG, CL, JH, ZL, WL, LL, PL, TY, SC, NL, JW, LN, MN, and MY analyzed data. TC, JR, BD, NL, ZZ, SL, MY, YZ, YW, JX, JH, ZL, RF, QC, LZ, and S-BG conducted the research and analyzed the results. TC, J-AC, RF, SY, JR, and BD wrote the manuscript. All authors read and approved the final manuscript.

## Funding

This study was partly supported by the Bill and Melinda Gates Foundation (INV-005834), Science and Technology Plan Medical and Health Project of Xiamen Science and Technology (No. 3502Z20194064), Talent highland special fund project of nanning (No. 2020021), Self-funded scientific research project of Guangxi Health Commission (No. Z20200786), National Natural Science Foundation of China (Nos. 11901027 and 11871093), China Postdoctoral Science Foundation (No. 2021M703426), and Pyramid Talent Training Project of BUCEA (No. JDYC20200327).

## Conflict of Interest

The authors declare that the research was conducted in the absence of any commercial or financial relationships that could be construed as a potential conflict of interest.

## Publisher's Note

All claims expressed in this article are solely those of the authors and do not necessarily represent those of their affiliated organizations, or those of the publisher, the editors and the reviewers. Any product that may be evaluated in this article, or claim that may be made by its manufacturer, is not guaranteed or endorsed by the publisher.

## Abbreviations

HIV: human immunodeficiency virus
AIDS: acquired immune deficiency syndrome
*R*_0_: basic reproduction number
*R*_*eff*_: effective reproduction number
ART: antiretroviral therapy
CDC: Centre for Disease Prevention and Control
SEITD: susceptible-exposed-untested HIV infection-tested HIV infection-dead
MSM: men who have sex with men.
